The article "Low Rates of Sustained Virologic Response with Peginterferon Plus Ribavirin for Chronic Hepatitis C Virus Infection in HIV Infected Patients in Rio de Janeiro, Brazil" was published in 2013. Journal: PLoS One.

# Low Rates of Sustained Virologic Response with Peginterferon Plus Ribavirin for Chronic Hepatitis C Virus Infection in HIV Infected Patients in Rio de Janeiro, Brazil

**DOI:** 10.1371/journal.pone.0067734

**Published:** 2013-07-09

**Authors:** Halime Silva Barcaui, Gerson Carreiro Tavares, Silvia Beatriz May, Carlos Eduardo Brandão-Mello, Márcia Maria Amendola Pires, Paulo Feijó Barroso

**Affiliations:** 1 Infectious Diseases Service, Department of Preventive Medicine, Hospital Universitário Clementino Fraga Filho, School of Medicine, Universidade Federal do Rio de Janeiro, Rio de Janeiro, Brazil; 2 Hospital Universitário Clementino Fraga Filho, School of Medicine, Universidade Federal do Rio de Janeiro, Rio de Janeiro, Brazil; 3 Hospital Gafree e Guinle, Universidade Federal do Estado do Rio de Janeiro, Rio de Janeiro, Brazil; Saint Louis University, United States of America

## Abstract

**Background:**

The standard treatment for chronic hepatitis C virus (HCV) infection in HIV-infected subjects is the combination of alfapeginterferon (PEG-IFN) plus ribavirin. We designed this study to evaluate the rate of SVR and predictors of SVR in a public health setting in Rio de Janeiro, Brazil.

**Methods:**

Retrospective cohort study of HCV/HIV co-infected patients treated with PEG-IFN plus ribavirin from 2004 to 2011 in 3 outpatient units in Rio de Janeiro. Exposure variables included age, sex, CD4+ cell count, HCV genotype, HCV and HIV viral loads, liver histology (METAVIR fibrosis scoring system) and previous treatment. The main outcome measurement was SVR.

**Results:**

100 patients were included in this analysis. Median age was 47 years and 68% were male. 80%, 4%, 14% and 2% were infected with HCV genotypes 1, 2, 3 and 4, respectively. At baseline, 77% had HCV viral load greater than 800,000 IU/ml, 99% had CD4+ greater than 200 cells/mm^3^ and 10% had a diagnosis of cirrhosis. The treatment was withdrawn in 9% of the subjects (5% with adverse effects and 4% dropped out). SVR was observed in 27 (27%) of the 100 patients included. 13 (13%) subjects were classified as null-responders, 33(33%) as non-responders, 9 (9%) as breakthrough and 9(9%) as relapsers. In the multivariate model only being infected with genotype 2 or 3 (p<0.01) and having low levels of gamma glutamyl transferase (GGT) at baseline (p = 0.04), were predictive of SVR.

**Conclusion:**

SVR in HCV/HIV co-infected subjects in a public health setting is similar to that observed in clinical trials, albeit very low. A delay in therapy initiation should be considered until new therapies as direct acting antiviral drugs (DAA) become widely available and tested in coinfected subjects.

## Introduction

Hepatitis C virus infection is a major cause of chronic hepatitis, cirrhosis and hepatocellular carcinoma, and is a leading cause of liver transplant in developed countries. HCV and HIV share similar routes of transmission and coinfection is common, being as high as 90% among intravenous drug users in certain geographic regions [1], [2].

HIV infection affects the natural history of HCV infection [3]. Coinfected subjects have higher HCV viral load and higher rates of HCV transmission when compared to HCV monoinfected [4]. In addition, increased prevalence of chronic hepatitis C and faster progression to cirrhosis is seen in these subjects [5], [6]. In the era of highly active antiretroviral therapy (HAART), coinfection has emerged as one of the major concerns for those caring for patients living with HIV [7]–[9].

The standard treatment for chronic HCV infection in HIV infected subjects is the combination of PEG-IFN plus ribavirin for 48 weeks. The rate of sustained virologic response: (SVR: HCV RNA below detection levels six months after treatment interruption using polymerase chain reaction assays), varies between 14–38% of those infected with HCV genotype 1 or 4 and 44–73% of those infected with genotypes 2 or 3 as observed in large international clinical trials [10]–[12]. There are scanty data evaluating HCV treatment responses among HIV-infected subjects in developing countries.

The aim of this study was to assess the rate of sustained virologic response and its predictors in a cohort of HIV and HCV coinfected subjects in Rio de Janeiro, Brazil.

## Methods

### Ethics Statement

The study protocol was approved by the institutional review board of the 3 institutions: Hospital Universitário Clementino Fraga Filho/Universidade Federal do Rio de Janeiro; Hospital Federal dos Servidores do Estado; Hospital Gafree e Guinle, Universidade Federal do Estado do Rio de Janeiro, Rio de Janeiro. Written consent was obtained from participants.

### Study Design, Setting and Study Population

This was a retrospective cohort study conducted from January 2004 to January 2011 at outpatient units of three tertiary hospitals in Rio de Janeiro: Hospital Universitário Clementino Fraga Filho of the Universidade Federal do Rio de Janeiro (HUCFF-UFRJ), Hospital Federal dos Servidores do Estado (HFSE) and Hospital Universitário Gaffrée e Guinle of the Universidade Federal do Estado do Rio de Janeiro (HUGG-UNIRio). HIV-HCV coinfected subjects, older than 18 years of age, that had been treated with the combination of PEG-IFN plus ribavirin during the study period in the three hospitals were included in the study. Subjects were excluded if they had evidence of hepatitis B coinfection. According to Brazilian guidelines the treatment period was defined as 48 weeks. Study personnel had no input into treatment decisions.

### Study Variables and Outcomes

The main outcome variable was sustained virologic response. Data on the frequency of null responders (failure to reduce HCV RNA by 2 logs after 12 weeks of therapy), breakthrough (reappearance of detectable HCV RNA in serum while still on therapy), non responders (failure to clear HCV RNA from serum after 24 weeks of therapy), and relapsers (reappearance of HCV RNA after end of treatment response) were collected.

In addition, data on early virologic response (EVR), rapid virologic response (RVR) and end of treatment response (EOT), when available, were also collected. A complete EVR was defined as HCV RNA below detection levels and a partial EVR was defined as a reduction in HCV RNA greater than 2 log_10_ by week 12 of treatment. Rapid virologic response was defined as HCV RNA below detection levels after four weeks of treatment and end of treatment response was defined as HCV RNA below detection levels when the treatment was completed.

Data on demographic, clinical and laboratory exposure variables were collected and included: age, gender, HAART use and regimen, CD4 cell lymphocyte count, HIV-1 plasma viral load, HCV genotype, baseline HCV RNA viral load, liver histopathology (as classified by METAVIR fibrosis scoring system) [13]. TSH, free T4, and liver enzymes. In addition, data on previous treatment with standard interferon and ribavirin were assessed. The reported reasons for treatment dose reduction and/or interruption during and at the end of the treatment were also collected. HCV and HIV viral loads were measured in blood samples using commercial immunoassays according to manufactureŕs recommendations. The lower detection limit for HCV- viral load in the assays used ranged from 9.6 IU/mL to 200 IU/mL. The lower detection limit of HIV-1 viral load ranged from 40 to 400 copies/mL.

### Data Collection and Statistical Analysis

Clinical and laboratory data were recorded in case report forms and entered in the SPSS© 17.0 software. The main outcome measurement was SVR. Exposure variables as HIV-1 viral load, HCV viral load and CD4+ lymphocyte counts were analyzed as continuous variables or were categorized when appropriate. The main analysis assessed the frequency of and factors associated with sustained virologic response. Univariate analyses were performed using x^2^ or Fisher exact test for categorical variables, and Student t test or Wilcoxon test for continuous variables as appropriate. Odds ratios (OR) and 95% CIs were calculated. Variables with p value <0.20 in the univariate analysis were included in the multivariate analyses to identify baseline predictors of SVR. We used a stepwise backward approach to assess factors independently associated with the main outcome. All reported *p* values are 2-sided.

## Results

### Study Population

One-hundred subjects were included in this analysis. Table 1 presents main demographic and clinical characteristics of the included subjects. Mean age was 47 years (range 20–70), and 68 (68%) subjects were male. Mean alanine transaminase (ALT) and gamma glutamyl transpeptidase (GGT) levels were 79 U/L (16–270 U/L) and 179 U/L (21–885 U/L), respectively. Mean platelets count was 197,313/mm^3^ (73,000–378,000/mm^3^). Mean albumin and bilirubin levels were 4.2 g/dL (3.2–5.4 g/dL) and 1.0 mg/dL (0.1–7.1 mg/dL), respectively.

**Table 1:** Baseline characteristics of the subjects (n = 100).

Mean age in years	47
Male sex (%)	68 (68%)
Median CD4 (cells/mm3) ± SD	500±192.7
HIV-1 Viral load below the lower detection limit (%)*	77/98 (79%)
Use of HAART (%)	89 (89%)
HCV Genotype 1	80 (80%)
HCV therapy naïve subjects (%)	80 (80%)
HCV viral load >800,000 IU/Ml** (%)	46/60 (77%)
Cirrhosis*** (%)	9/88 (10%)

HAART: Highly active antiretroviral therapy; HCV: Hepatitis C virus.

* Available for 98 subjects.

** Available for 60 subjects.

*** Liver histopathology available for 88 subjects (METAVIR Fibrosis scoring system).

HCV genotype 1 was present in 80 (80%) of the patients. Among these subjects, 24 subjects were classified as genotype 1a and 15 as genotype 1b. In 41 subjects no specific subtype could be characterized. Genotypes 2, 3 and 4 were observed in 4 (4%), 14 (14%) and 2 (2%) of the subjects, respectively. Eighty (80%) of the subjects were HCV treatment naïve. Twenty subjects had a history of previous treatment with standard interferon and ribavirin. Nineteen (95%) of these previously treated subjects was classified as non-responders and one patient did not complete the treatment due to hematologic toxicities. Baseline HCV viral load data was available for 60 (60%) subjects. Among these, 44 (77%) had HCV viral load above the upper limit of detection (800,000 IU/mL). Baseline liver histopathology was available for 88 (88%) subjects. According to METAVIR fibrosis scoring system, 9 (10%) subjects were classified as having cirrhosis. Three (3%), 37 (42%), 28 (32%), 11 (13%) were classified as having fibrosis stages 0, 1, 2 and 3 respectively. PEG-IFN 2a was prescribed for 62 (62%) subjects and IFN 2b was prescribed for 38 (38%).

Median baseline CD4+ lymphocyte count was 495 cells/mm^3^ (187–1941 cells/mm3) and 99 (99%) had CD4 count above 200 cells/mm3. Eleven patients (11%) were antiretroviral naïve and 89 (89%) were using HAART. 43 (48%) were using a protease inhibitor containing antiretroviral regimen and 48 (54%) a non-nucleoside containing HAART. HIV viral load was below detection levels in 77(87%) of the subjects on therapy.

### Virologic Response

The sustained virologic response was observed in 27 (27%) subjects. Five subjects (5%) had the treatment suspended due to hematological toxicity (3 with genotype 1 and 2 with genotype 2 or 3) and 4 (4%) subjects dropped out (all were genotype 1). Forty five (45%) subjects completed the 48 week treatment regimen (11 with genotype 2 or 3 and 34 with genotype 1 or 4) and treatment was discontinued before 48 weeks in the remaining 46 subjects because of null response or non response. Thirty-six (36%) subjects had an HCV-PCR below detection levels at the end of treatment. Nine (25%) of these subjects relapsed. Relapses were observed in 9% (1/11) of the subjects infected with genotype 2 or 3 and 32% (8/25) of the subjects infected with genotype 1 or 4.

At the end, 13 (13%) subjects were classified as null-responders, 33 (33%) as non-responders, 9 (9%) as breakthrough and 9 (9%) as relapsers. Among patients with genotypes 2 or 3 (18%), one subject was a null responder (5%) and 5 were non responders (28%) and among those with genotype 1 or 4, 12 were null responders (15%) and 28 were non responders (34%).

SVR was observed in 15 (19%), 2 (50%), 8 (57%) and 2 (100%) of the subjects with genotypes 1, 2, 3 and 4 respectively (p<0.01, chi square test).

### Predictors of Virologic Response

#### Univariate analysis

The distribution of main exposure variable values in relation to SVR is presented in Table 2. Mean age and gender distribution was not associated with SVR. Among baseline liver function tests and complete blood count only GGT levels were statistically associated with SVR. Subjects with SVR had lower values of GGT. (111 IU/mL in individuals with SVR and 204 IU/mL in those without SVR, p<0.01). Variables related to HIV infection were not associated with SVR. Those who achieved SVR had a median CD4+ count of 537 cells/mm^3^ as opposed to a median of 488 cells/mm^3^ in those who did not achieve SVR (p = 0.29). SVR was observed in 20 (26%) subjects with HIV-1 viral load below detection levels and in 6 (33%) among those with detectable HIV-1 viral load (p = 0.87). SVR was not observed in any of the 3 subjects with HIV-1 viral load above 50,000 copies/mL.

**Table 2:** Association of selected baseline variables with sustained virologic response (SVR).

	Subjects with SVR	Subjects without SVR	*P* value
**Mean age**	47	47	0.84
**Male sex (%)**	19 (68%)	49(72%)	0.81
**Infected by HCV genotype**, **1 or 4 (%)**	17 (21%)	65 (79%)	0.01
**Cirrhosis present, (%)**	3 (33%)	6 (67%)	0.67
**Mean CD4+ lymphocyte count** *	631	548	0.29
**HCV viral load,** **>800.000** **IU/mL (%),**	14 (30)	32 (70)	0.71
**Albumin(g/dL)** *	4.3	4.2	0.11
**Mean Platelets (mm^3^)** *	184,704	202,041	0.17
**Mean GGT (IU/mL)** *	111	204	<0.01
**Mean ALT(IU/mL)** *	86	76	0.74
**Mean Bilirubin** * **(mg/dL)**	0.8	1.0	0.13

HCV: Hepatitis C virus; GGt: Gamma glutamyl transferase; ALT: Alanine transaminase.

* available for all (100) subjects.

Among exposure variables related to HCV infection and therapy only HCV genotypes and early virologic responses were associated with SVR. Subjects with genotypes 2 or 3 had a greater probability of SVR. Ten (56%) of those infected with genotype 2 or 3 had an SVR as opposed to 17 (21%) of those infected with genotypes 1or 4 (p<0.01). Fifty nine (59%) sujects had early virologic response evaluated. SVR was observed in 17 (61%) subjects with complete EVR as opposed to 1 (8%) of those subjects with partial ERV ((p<0.01).

Baseline HCV viral load, METAVIR fibrosis scoring system and previous treatment were not associated with SVR. SVR was observed in 1 (33%), 12 (32%), 5 (18%), 3 (27%) and 3 (33%) of the subjects with METAVIR fibrosis scoring system grades 0, 1, 2, 3 and 4 respectively (p = 0.78).SVR was observed in 4 (20%) of previously treated subjects in contrast to 23 (29%) of HCV treatment naïve (p = 0.58). Type of PEG-IFN had no association with SVR. Users of PEG-IFN 2a had an SVR of 29% (11/38) while those using PEG-IFN 2b had an SVR of 26% (16/62), p = 0.82.

#### Multivariate analysis

Table 3 shows the final multivariate logistic model. Being infected with HCV genotype 2 or 3 (OR: 4.9; p<0.01; 95% CI: 1.6–15) and lower levels of GGT at baseline (OR: 1.01; p = 0.04) were independently associated with a sustained virologic response.

**Table 3:** Predictors of Sustained virologic response – Multivariate analysis.

Variable	OR (95% CI)	p value
**HCV genotype 2 or 3**	4.9 (1.6–15)	<0.01
**Mean GGT levels (IU/mL)**	1.01 (1–1.01)	0.04

HCV: Hepatitis C virus; GGt: Gamma glutamyl transferase.

OR (95% CI): Odds Ratio (95% confidence interval).

### Adverse Events and Treatment Modifications

Four patients (4%) dropped out. Among the remaining 96, dose modification of interferon, ribavirin or both was needed in 29 (30%) subjects. Treatment was discontinued in 5 (5%) individuals due to hematological toxicity. Erythropoietin and filgastrim were not available for these 5 subjects. Filgastrin was used by 11 (11%) of the subjects and erythropoietin by 3 (3%) Ribavirin dose was reduced in 25 (25%) subjects and interferon dose was reduced in 11 (11%) subjects. Seven (7%) subjects had doses of both drugs reduced. Among those requiring dose reduction only 4 (36%) and 2 (8%) had access and used filgastrin and erythropoietin, respectively.

The use of stimulating growth factors did not interfere with SVR.SVR was observed in 26 (27%) subjects who did not use erythropoietin and in 1 (33%) subject who used the drug (p = 1). Eleven subjects used filgrastim. SVR was observed in 3 (27%) of those who used this drug and in 24 (27%) of those who did not (p = 1).

## Discussion

In this population of HIV-infected subjects, in a resource-limited setting, the treatment of chronic HCV infection led to a sustained virologic response in only 27% of those subjects treated with peginterferon plus ribavirin. This proportion of SVR observed in outpatient units of the public health sector in Rio de Janeiro, Brazil, is similar to those reported in three clinical trials conducted in resource-rich countries^10–12^. Among subjects with the most prevalent genotype in this population, genotype 1, the rates of responses were even smaller. SVR in genotype 1 infected subjects was observed only in 19% of subjects. SVR was observed in 50, 57% and 100% of subjects infected with genotypes 2, 3 and 4 (2 subjects), respectively. These proportions are also in line with those reported in the cited trials ^10–12^, More recently conducted studies have observed SVR rates up to 35% in patients with genotype 1 when treatment in subgroups of patients is prolonged to 72 weeks [14].

Twenty-nine (30%) subjects required reductions of PEG-IFN, ribavirin or both because of treatment side-effects, either anemia or neutropenia. It is reasonable to hypothesize that an increased access to growth stimulating factors, such as erythropoietin and filgrastim, would change this scenario and fewer subjects would need to reduce the prescribed dose.

In Brazil, the anti-HCV drugs, PEG-IFN and ribavirin are available, for free, through specific Ministry of Health programs [15]. These programs, however, do not guarantee a prompt access to these growth stimulating factors. Interestingly, the SVR rate observed in this cohort did not change when reduction or suspension of the drugs were necessary, as previously reported by Tala et al [16]. These findings contrast with those that report that lower doses of ribavirin influence treatment outcome and from the studies that report that erythropoietin and filgrastim allows the maintenance of recommended doses of PEG IFN and RBV [17]–[23]. One possible explanation for these differences may be the fact that a small proportion of the participants of this cohort used one of these drugs.

Baseline CD4+ lymphocyte count, HCV and HIV viral loads, previous treatment and liver fibrosis were not predictors of SVR, as opposed to data that have been reported from large multi-center trials or single center studies [10]–[12], [17]. The high CD4+lymphocytes counts (median 500 cells/mm3) and the low frequency of advanced fibrosis (23%) observed in this cohort may explain these conflicting results. In line with other studies [24]–[28], subjects with complete early virologic response had an increased chance of achieving SVR (OR = 17, p<0.01).

The consistency of this finding in several studies may be considered in the management of coinfected subjects as an indication to evaluate treatment interruption on week 12 or the possibility to prolong treatment to 72 weeks in those who do not have a complete early virologic response [29].

Unfortunately, few clinicians had prompt access to laboratory results on week 12. An increased availability and prompt access to these results would be of great value to guide physicians in evaluating treatment interruption on week 12 (and avoiding unnecessary costs and toxicities) in those who do not have early virologic response.

In this cohort, being infected with genotype 2 or 3 and having lower gamaglutyltransferase levels were independently associated with SVR in the final multivariate model. The influence of HCV genotype on treatment response has been extensively reported in the literature [10]–[12]. The association of GGt levels with SVR has been observed in HCV monoinfected subjects, but not in those coinfected with HIV [30], [31]. The real clinical meaning and predictive value of this observation needs to be further studied.

One limitation of this study is retrospective cohort design. In addition, only 31 and 59 patients of this cohort had quantitative PCR results available at week 4 and 12, respectively. The lack of availability of these expensive tests and the lag time to obtain results in the clinical units may explain this limitation. This common scenario in resource-constrained settings may have determined extended treatments that would fail at the end, bringing increased costs and unnecessary toxicities.

In a resource-constrained setting, in a low income country, the rate of SVR observed was similar to those observed in multi-centric clinical trials conducted in high-income countries. Nevertheless, these rates are extremely low and a great proportion of this population was submitted to an expensive, toxic and prolonged drug regimen with no real benefit. Several new drugs to treat HCV have been developed in recent years [32]–[35]. Protease inhibitors for the treatment of genotype 1 HCV monoinfected patients have been approved by regulatory agencies in Brazil, North America and Europe [36]–[38]. Clinical trials evaluating direct acting antiviral drugs (DAA) in coinfected patients with HIV and HCV are ongoing and although drug interactions may be problematic, improvements in SVR rates are expected [39]–[41].

In summary, the decision to start treatment of HCV-HIV co-infected subjects with PEG-IFN and ribavirin needs to be extensively discussed with patients. Costs, side effects and low response rates have to be weighted against the anticipated delay to have new drugs available. In patients with genotypes 2 and 3, the decision to start the standard treatment with PEG-IF and ribavirin may be an easier one as this treatment is reasonably effective. The rate of SVR in subjects who completed 48 weeks of therapy and had an EOT were 91% among subjects with genotype 2 or 3. In contrast, for subjects with genotype 1 HCV infection, especially those with unfavorable IL28B genotype, who have failed previous treatment and have mild to moderate fibrosis, waiting for the alternative therapies may prove to be a better decision.
